The article "Transition in Dental Treatment Utilization in Jammu And Kashmir, India - A 10 Year Retrospective Study" was retracted in 2017. Reason: fabricated or falsified data.

#  Transition in Dental Treatment Utilization in Jammu And Kashmir, India - A 10 Year Retrospective Study 

**DOI:** 10.3126/nje.v6i4.17257

**Published:** 2016-12-31

**Authors:** Aasim Farooq Shah, Manu Batra, A. Ishrat

**Affiliations:** 1 Registrar, Department of Public Health Dentistry, Government Dental College and Hospital Shreen Bagh, Srinagar, Jammu and Kashmir, India. 190010.; 2 Assistant Professor, Department of Community and Preventive Dentistry, UCMS College of Dental Surgery Bhairahawa, Nepal.; 3 Dental Surgeon [School Health Program], J&K Government Health Services. Srinagar, Jammu and Kashmir India 190001

**Keywords:** Utilization Trend, Dentistry, Behaviour, Restorative Dentistry, Oral health.

## Abstract

**Background:**

Utilization of health services is the actual attendance by the members of the public at health care facilities to receive care. Utilization, serves as an important tool for oral health policy decision-making. The aim of the present study was to retrospectively gauge and assess the utilization pattern of the dental treatments which was given in hospital for last 10 years.

**Materials and Methods:**

This retrospective infirmary based study was carried out at Sheri Kashmir Institute of Medical Sciences (SKIMS), Srinagar, Jammu and Kashmir, India. The yearly outpatient department (OPD) records for the utilization of specific dental treatment of a total of 103963 patients were assessed retrospectively from 2014 to 2003. Trend analysis was used to assess the trend of utilization of each speciality with best fitted linear trend lines.

**Results:**

The pattern of new patients has also shown a constant rise during the study period except for 2008 and 2009. The utilization of oral surgery speciality has shown a tremendous fall from 2003 to 2014 whereas the number of patients coming to periodontics and conservative dentistry has shown an increasing pattern.

**Conclusion:**

Utilization of oral health care has long been used as an indicator of oral health related behaviour of a population. In the present study it can be conclude that the outlook of the population under study has changed from blood and vulcanite dentistry outlook and is moving towards restorative dentistry. .

## Introduction

Health has been at the centre of human concern since ancient times. The practice of medicine has come a long way since the time of magic, religion and supernatural thoughts to a modern science following evidence-based practice with a range of services extending from preventive, promotive, curative to rehabilitative offered to the individual and community. 

 Utilization of health services is the actual attendance by the members of the public at health care facilities to receive care. Utilization, which measures the number of visits per year or the number of people with at least one visit during the previous year, serves as an important tool for oral health policy decision-making [ 1 ]. As described in the recent World oral health report 2003 oral diseases have a considerable impact on individuals and communities, as a result of the pain and suffering, impairment of function and reduced quality of life that they impose [ 2 ]. 

 Dental care utilization can be defined as the percentage of the population who access dental services over a specified period of time [ 3 ]. Utilization of any type of health care is a complex phenomenon and multifaceted human behaviour. Various theories and conceptual models have been proposed to explain this phenomenon. The determinants of oral health care can be classified as predisposing (socio demographic factors like age, sex, occupation, and social network), enabling (transportation, income, and information), and need (perceived health or professionally assessed illness) factors [ 4 ]. 

 Oral treatment seeking behaviour refers to the behaviour of seeking professional help to curb symptoms presenting like pain, bleeding, swelling, bad breath, developmental anomalies, mobile teeth, ulcer, caries, sensitivity and fractured teeth. Dental disease is a serious public health problem with universal distribution and affecting all age groups [ 5 ]. Oral treatment seeking behaviour is greatly influenced by various factors which can be related to the cost of treatment, accessibility to health facility, time factor, level of education knowledge of oral diseases and severe symptoms such as pain tend to influence treatment seeking behaviour more than other factors. 

 Barriers to seeking oral health treatment like ignorance, lack of awareness, high cost of treatment, inaccessibility to oral health facility and lack of time also play a significant role. However in recent years it has been observed that the attendance at the health centres have considerably improved. This increase in the utilization of the health services can be attributed to the increase in the level of awareness and education in the masses. Many studies have been conducted on the utilization of the dental health services in various countries including India [ 6, 7 ]. The results have shown a considerable increase in the utilization of dental services.

However the studies on the pattern of the given treatment have not been performed. It becomes imperative on us to know the felt need of the patients when it comes to their utilization of dental services. Unless it is not assessed that what type of the treatment population is asking for in a health centre we cannot assess the level of education or whether the appropriate knowledge has been imparted to the population or not. Shift from ancient trends of treatments to the modern types of treatments shall be assessed in order to improve the patient education as well as the system which is responsible for the health education. A shift from "blood and vulcanite" dentistry to the modern restorative dentistry if present needs to be assessed and if not present needs to be created [ 8 ]. Thus there is need to undertake studies which focus on the changes in the development of dental treatment patterns among people by gauging utilization rates. 

 In the state of Jammu and Kashmir, India most services are paid entirely by the patients themselves, and most commonly delivered by private practitioners. Thus information on dental conditions, treatment needs and habits have been sparse. The aim of the present study was to retrospectively gauge and assess the utilization pattern of the dental treatment which was given in a SKIMS hospital, Srinagar from 2003 to 2014 with a primary objective to access the change in the trend of utilization of restorative dental procedures as compared to oral surgical procedures.

## Methodology

### Study Design and the Participants:

This retrospective infirmary based study was carried out at SK Institute of Medical Sciences, which is located in Srinagar, the summer capital city of Jammu and Kashmir state, 10 km from central business centre. It is the largest hospital in Kashmir and provides treatment of dental conditions. The yearly outpatient department (OPD) records for the utilization of specific dental treatment at the dental wing from 2003 to 2014 were analysed retrospectively. All the patients whose records were present in the hospital database during this period for any type of dental treatment were included.

### Data Collection:

Records of a total of 103963 patients who had visited from 2014 to 2003 were assessed retrospectively. Out of the total number of the patients 45273 patients were revisit cases throughout this time period. The number of the new patients who had visited during this period was 58690. Data was collected in for of hospital records for all these patients.

### Inclusion Criteria:

All the patients who had visited the outpatient department (OPD) for the utilization of any kind of dental treatment at the dental wing of SK Institute of Medical Sciences, from 2003 to 2014 were analysed retrospectively.

### Exclusion criteria:

Records of those patients who had been referred to some other department or hospital for specialized treatments as major surgical procedures or patients with oral cancer who were not treated at the dental wing of SK Institute of Medical Sciences were excluded from the study. From the study.

### Sample size calculation:

Records of a total of 103963 patients who had visited from 2014 to 2003 were assessed retrospectively. All the records which were pertaining to the Dental wing of the hospital were assessed and the data was analysed retrospectively for all these records.

### Outcome Variable:

The present study assessed the change in the perception in the utilization pattern of the dental treatment in a retrospectively selected population for a period of 12 years.

### Explanatory variable:

The influx of patients each year was segregated into new and recalls categories. The various dental treatments were classified under specialities i.e. oral surgery, periodontics, conservative dentistry and prosthodontics. This study assessed the change in the utilization pattern of different dental treatments by the population retrospectively.

### Ethical committee approval:

The ethical clearance was taken from the ethical board of the SK Institute of Medical Sciences, Srinagar. The data was analysed in a most professional manner keeping in view the ethics and confidentiality of the patient records.

### Data management and statistical analysis:

Data were entered into Microsoft excel software and exported to SPSS Version 15 for analysis. Descriptive statistics was used to report the frequency and percentage of independent variables. Trend lines analysis with best fitted linear trend lines was used for judging the difference in the patient referrals with time.

## Results

The current study was conducted in dental wing of SK Institute of Medical Sciences, Srinagar, India. The patient data records of 12 years, from 2003-2014 were assessed. Table 1 and Graph 1 present the patient influx or total number of the patients who had visited the dental wing in each year from 2003 to 2014. There was a steady increase in number of overall patients except for 2008 and 2009 which have showed a slight fall in numbers. The proportion of new patients has also shown a constant rise during the study period. Table 1 also presents the number of referrals to various sections within the dental wing. An increase in the conservative treatment is obvious from year 2003 to 2014. Pattern of utilization of specialized dental care services during the study period is plotted in Graph 2 The utilization of oral surgery speciality has shown a tremendous fall from 2003 to 2014 whereas the number of patients coming to periodontics and conservative dentistry has shown an increasing pattern. Patients being referred for prosthodontic care also showed a steady increase Graph 3 and Graph 6 present the trend line of different treatments. The trend of the fall of percentage of patients visiting oral surgery department is evident in Graph 3 However Graph 4 to Graph 6 show gradual rise in percentage of patients visiting periodontics, conservative dentistry and prosthodontics.

## Discussion:

Dental disease as dental caries and periodontal diseases is a serious public health problem in whole of the world and are prevalent in all age groups. However, despite of their universal distribution only a few people seek dental care or utilize it. There exists a wide gap between the actual dental needs of the population and the demand for dental care which is quite clear from the past cited literature. The barriers in the utilization of the dental care can be removed by motivating people by making them aware about the oral health problems and removing anxiety and fear so that they develop positive attitude towards dental treatment. Previous studies have revealed that the high cost of oral health care and fear of dentists or dental instruments have been major barriers for seeking oral care [ 9 ]. 

 Increasing Awareness 

 Though the present study shows an increase in the number of the patients who seek dental treatment in the dental section of the SK Institute of Medical Sciences, there is a clear difference in the influx of the patients from 2003 to 2014. Records of a total of 1, 03,963 patients who were assessed retrospectively comprised of 58690 new patients while 45273 patients were revisit cases throughout this time period. There has been a steady increase in the number of the new patients every year. This trend shows that there has been an increase in the oral health awareness during this time span which has led to the increase in the patient influx. Some earlier studies have also reported an increase in the number of the patients in the dental hospitals [ 8 ]. 

 Change in perception: 

 Findings from the present study support the assumption that, in developing countries, visits to dental-care services are usually carried out because of agony caused by dental pain. Many previous studies have revealed that the high cost of oral health care have been the major barriers for seeking oral care [ 9 ]. The increased number of the patients in the section of oral surgery in the earlier part of the study period denotes that patients were usually opting for blood and vulcanite dentistry. This observation is in accordance with those of previous studies conducted in the United Republic of Tanzania [ 10 ] and Srilanka [ 11 ].

Previous studies have shown that the younger age group visit dentist more regularly in comparison to the older age group which may be due to the fact that the younger age group had more knowledge and fewer barriers in seeking dental care [ 12 ]. Syrjala et al. also found that the older age group did not think that oral health was important which may be true for the older group. However in the present study stratification of the data was not possible for the gender or any other variables. The main finding which comes forward in the present study is that an increase in the demand in the restorative services can be seen in the sample population. In the Western countries, the demand for dental care is gradually growing, although utilization rates differ between countries [ 13, 14 ]. 

 This development should probably be seen in perspective with modernistic standards and stereotypies as good health, young and slim body, brown face and nice shiny white teeth. The reasons for seeking dental care include several basic wishes of physical, psychological and social origin such as chewing ability, feeling fit dentally and comfortable and overall being good-looking and having a pleasant smile. 

 Change in Utilization pattern: 

 However, in present study the trend towards the preventive and restorative dentistry shows an increase with each passing year. People have opted periodontic and conservative procedures more often than the oral surgical procedures as dental extractions. The trend analysis shows that there has been an increase in the procedures as scaling and restorative dentistry from 2003 towards 2014. This trend has been shown in various developed countries in the world [ 15 ]. 

 Possible reasons for this increase in the demand of the dental health services in the study population can be increase in the education level of the population; increase in the socio economic status or increase in the awareness about oral health. This information can help dentists and planners how to optimally distribute resources viz., manpower and money and produce the greatest amount of additional benefits. This also suggest that Dental surgeons and dental health workers have been playing their role adequately in facilitating public enlightenment and people have appreciated the need for regular dental care by utilizing the services. 

 Many previous studies have revealed that the high cost of oral health care and fear of dentists or dental tools have been the major barriers for seeking oral health care [ 9 ] . Patient education is must and shall gradually bring such intuitions down. It is also important to remove the barrier of high cost of healthcare by conducting free oral health examination camps, which can be proved to effective in screening for diseases and for providing preventive care. 

 Utilization of oral health care is an indicator of oral health behaviour of a population, with underlying social determinants. Since high costs one of the main barricades to utilization of oral health care, social and economic up-liftment through policies addressing the issues of sickness and rehabilitation benefits, child benefits, healthcare facilities, and women empowerment is crucial for the successful delivery of oral health services.

It shall also be highlighted that the impact of health insurance coverage can also drastically help people to go for dental services at an earlier stage. However the dental health insurance is practically not available in this part of the country but it shall be made available as soon as possible to keep the present trend increasing.

## Conclusion

Utilization of oral health care has long been used as an indicator of oral health related behaviour of a population. In the present study it can be concluded that the outlook of the population under study has changed from blood and vulcanite dentistry outlook and is moving towards restorative dentistry. This can be enough for the planners to focus the resources towards the proper direction or the felt needs of the population.

### Limitations of the study

The present study has been a retrospective study where the records of a hospital have been used for making the results. Certain limitations may surface within the records as stratification according to the gender, age and socio economic status could have been more informative as to which group or social class had used the treatment more often. Other limitation is that it may cover only the catchment areas of the hospital and not the whole of the population of the state or the country. The presence of the staff pattern in the dental section of the hospital has almost remained the same all throughout the period of the study thus that could have a little effect on the outcome of the study.

### Future scope of the study:

Studies regarding the utilization dental services by north.east Indian population are almost non.existent. Therefore it is the responsibility of the health professionals of to gather the data on the utilization of dental services by people residing in this part of the country.

### What is already known on this topic:

The truth that dentistry has changed with passing years is not unknown. There have been changes in the insight of the dentists and similarly the treatments have become much sophisticated and contemporary. It has been witnessed that there has been an increase in the utilization of the dental services in developing countries but the pattern of this utilization has not been investigated in depth.

### What this study adds:

The present study presents the information about the population’s use of dental services. It is both necessary and useful as the dental sector experiences the impact of changing forces which influence the number of people who visit the dentist and the type of services they consume. When such information is available, it can help dentists and planners more toward more optimal distributions of manpower and money

## Figures and Tables

**Graph 1:** Graph 1: Distribution of new and revisit appointments during 2003-2014 time period.

**Graph 2:** Graph 2: Distribution of referral of patients during 2003-2014 time period.

**Graph 3:** Graph 3: Trend line showing variation of referrals to oral surgery department.

**Graph 4:** Graph 4: Trend line showing variation of referrals to periodontics department.

**Graph 5:** Graph 5: Trend line showing variation of referrals to conservative dentistry department.

**Graph 6:** Graph 6: Trend line showing variation of referrals to prosthodontics department.

**Table 1:** Table 1:Patient influx in dental wing during 2003-2014 time period with number of referrals.

**YEAR**	**New patients**	**Revisit Patients**	**Referrals**	**Oral surgery**	**Periodontics**	**Conservative**	**Prosthodontics**	**TOTAL**
2003	3963	3430		1405	321	695	300	**7393**
2004	4658	2570		1330	460	844	361	**7228**
2005	5101	5213		1932	1153	936	537	**10314**
2006	5312	4558		2033	612	1153	225	**9870**
2007	4839	4176		1389	763	1298	543	**9015**
2008	4570	3293		1581	612	1216	145	**7863**
2009	3672	3109		1304	684	1387	108	**6781**
2010	5176	3954		1496	1283	1411	488	**9130**
2011	4589	3654		1243	1253	1679	365	**8243**
2012	5931	3792		1309	654	1412	687	**9723**
2103	5267	3525		1479	892	1603	252	**8792**
2014	5612	3999		1465	1105	1409	491	**9611**
Total	**58690**	**45273**		**17966**	**9792**	**15043**	**4502**	**103963**
